The article "Double-Balanced Loss for Imbalanced Colorectal Lesion Classification" was published in 2022. Journal: Comput Math Methods Med.

# Double-Balanced Loss for Imbalanced Colorectal Lesion Classification

**DOI:** 10.1155/2022/1691075

**Published:** 2022-08-08

**Authors:** Chang Yu, Wei Sun, Qilin Xiong, Junbo Gao, Guoqiang Qu

**Affiliations:** ^1^Information Engineering College, Shanghai Maritime University, Shanghai 201306, China; ^2^Department of Gastroenterology, Eastern Hospital, Shanghai Sixth People's Hospital, Shanghai 201306, China

## Abstract

Colorectal cancer has a high incidence rate in all countries around the world, and the survival rate of patients is improved by early detection. With the development of object detection technology based on deep learning, computer-aided diagnosis of colonoscopy medical images becomes a reality, which can effectively reduce the occurrence of missed diagnosis and misdiagnosis. In medical image recognition, the assumption that training samples follow independent identical distribution (IID) is the key to the high accuracy of deep learning. However, the classification of medical images is unbalanced in most cases. This paper proposes a new loss function named the double-balanced loss function for the deep learning model, to improve the impact of datasets on classification accuracy. It introduces the effects of sample size and sample difficulty to the loss calculation and deals with both sample size imbalance and sample difficulty imbalance. And it combines with deep learning to build the medical diagnosis model for colorectal cancer. Experimentally verified by three colorectal white-light endoscopic image datasets, the double-balanced loss function proposed in this paper has better performance on the imbalance classification problem of colorectal medical images.

## 1. Introduction

A survey shows that malignant tumors have become the first killer of Chinese residents' health by 2020. There is an evidence that the incidence rate and mortality of colorectal cancer are increasing at a particularly significant rate. In 2020, the number of new cases and deaths of colorectal cancer has increased to more than 500,000 and more than 300,000, respectively, which has seriously threatened the health of Chinese residents [1]. Colorectal white-light endoscopy is one of the most widely used of polyp detection and have been extensively used for early colorectal cancer screening. Previous research has shown that missed and misdiagnosed colorectal polyps will increase the possibility of colorectal cancer, and their survival rate is less than 10% [2]. Therefore, the proper classification of colorectal polyps by white-light endoscopic images can be used to assist physicians in the early screening of colorectal cancer.

With the application of artificial intelligence in the field of intelligent medicine, deep learning models are widely used in the lesion detection and classification of medical images. This paper reviews and compares the main research work of large intestine white-light endoscope image recognition from two aspects: deep learning models and lesion classification methods; the results are shown in Table 1. The existing body of research on colorectal polyps' classification suggests that classification standards are not uniform. Komeda et al. [3, 4] used convolutional neural networks to classify lesions into neoplastic and nonneoplastic and adenomatous and nonadenomatous. Gao et al. [5] used ResNet50 [6] to distinguish whether colonoscopic images contain lesions, then detected specific lesions and divided them into adenoma, cancer and polyp, which detected AP50 up to 0.903. Taş and Yilmaz [7] proposed to perform super-resolution reconstruction of colonoscopic images to obtain high-resolution images, then use Faster R-CNN [8] for detection, which improved the accuracy of model detection by 8% through super-resolution processing. Shin et al. [9] used image enhancement such as rotation and scaling to increase the number of training samples and then used Faster R-CNN for detection. Shin et al. [10] proposed a framework for generating synthetic polyp images to augment the training data to detect polyps using Faster R-CNN with a 20% improvement in accuracy. Among them, the literature [7, 9–11] did not classify the lesions but only detected the presence of polyps.

In early colorectal cancer screening, the classification of colorectal polyps is important. Clinically, physicians need to determine whether to perform resection surgery based on the specific category of polyps. At present, there is little research on the classification of colorectal polyps under deep learning, mainly due to the lack of large public datasets for polyp classification [11]. Based on the experience of doctors in the Shanghai Sixth People's Hospital (East Hospital) in the clinical diagnosis of colon white-light endoscopy, this paper adopts the classification criteria proposed in literature [4]; that is, colon lesions are divided into polyps (polyp), adenomatous polyps (adenoma), and cancerous structures (cancer). Furthermore, the collected colorectal images with lesions were labeled into three categories to carry out a classification study of colorectal white-light endoscopic images.

## 2. Problem Statement and Background

In recent years, deep learning has achieved good results in the detection and classification of medical image lesions, which can assist doctors in the diagnosis and treatment work to a certain extent. This mainly depends on the powerful learning ability of deep learning models in the image field and the recognition accuracy that can match or even exceed the human eyes. However, the deep learning model is based on the assumption that the samples are independently and equally distributed in the training set, but this premise does not hold in most medical image datasets. A survey showed that about 75% of colorectal polyps are adenomatous polyps [12], which leads to the fact that most of the colorectal white-light endoscopic images collected by doctors from clinical diagnosis are adenoma images. Unbalanced data makes it difficult for deep learning models to be applied in the field of medical-assisted diagnosis. There are two types of approaches designed to address imbalance classification. The first category is the data-level approach, which adjusts the adaptability of the model to the data by changing the data distribution of the training set, such as random oversampling and random undersampling. The second category is the algorithmic-level approach, which does not change the training set but adjusts the training strategy or model structure, such as reconfiguring the classifier, two-stage training, and improving the loss function. Moreover, methods that combine the two types are available.

### 2.1. Data-Level Approach

Random undersampling and random oversampling are the classical methods to solve data imbalance; both of them change the original distribution of the dataset. In 2015, Bae and Yoon [13] proposed an upsampling enhancement framework based on data sampling to use rebalanced datasets to learn comprehensive classifiers and use them to detect different types of polyps. The experimental results show that the performance is improved compared with other most advanced detectors. However, random undersampling may cause the samples to lose important feature information during undersampling, while random oversampling increases the risk of overfitting. SMOTE [14] is a more advanced sampling method to overcome this problem, in which new samples are generated by adding data points from the nearest neighbors by interpolation; the limitation of this method is that it cannot overcome the problem of data distribution in unbalanced datasets, which increases the difficulty of classification algorithms to classify them. Another sampling method is class-aware sampling for stochastic gradient descent optimization neural networks [15], whose main idea is to ensure that the sample classes of each batch are evenly distributed in training.

### 2.2. Algorithm-Level Approach

One algorithm-level approach to address data imbalance is to reconfigure the classifier, which can be implemented in various ways, such as one-class classifier, which uses small classes as outliers and transforms the classification problem into abnormal detection [16]. Two-stage training [17] is first performed on a balanced dataset, and then, the final output layer is fine-tuned on the unbalanced original dataset. Although these methods can alleviate the data imbalance problem to some extent, the improvement of loss function has more attractive features, such as ease of implementation. Cross-entropy loss is widely used in classification problems, but it cannot handle data imbalance. A simple improvement is to use weighted cross-entropy (WCE) according to the number of categories, which is often ineffective in practice. In 2019, Cui et al. [18] proposed the class-balanced loss framework, using the effective number of samples per class to inversely weight the loss, and this method can effectively solve the class number imbalance problem. Kim et al. [19] proposed complement cross-entropy (CCE) to solve the problem of imbalanced classification and proved that suppressing the probability of the error class helps the deep learning model to learn discriminative information. By neutralizing the confidence of the error sample, the minority class samples get more learning opportunities. In addition, the sample difficulty imbalance can be handled by improving the loss function. In 2016, Shrivastava et al. [20] proposed the OHEM algorithm to screen out difficult samples based on the loss value of the input samples, and then, the screened samples are applied to training in stochastic gradient descent. This method achieves online hard example mining, but it completely discards simple samples, which leads to the model's inability to improve their detection accuracy. In 2017, Lin et al. [21] proposed focal loss to increase the model's focus on difficult samples by dynamically adjusting the loss contribution of difficult samples by introducing a (1 − *p*)^*γ*^ modulation factor in the cross-entropy, but this approach assigns high weights to outliers as difficult samples. The GHM [22] loss function can improve this problem, and its basic idea is to start from the gradient parity of the samples and to dynamically weight the samples according to the proportion of samples accounted for by the gradient parity so that easy samples with small gradients are downweighted, difficult samples with medium gradients are upweighted, and outlier samples with large gradients are downweighted.

## 3. Materials and Methods

### 3.1. The Proposed Methods

The most common loss function used in deep learning multiclassification tasks is cross-entropy (CE) loss. The cross-entropy loss gives equal importance to each data instance, which will lead to the network monitoring the classes with fewer number of observations. Therefore, CE loss is inappropriate in classification tasks under class imbalance. This paper proposes a new loss function named double-balanced (DB) loss. We derive it from the perspective of sample size and sample difficulty.

#### 3.1.1. Imbalance of Sample Size

Usually, the method to deal with the unbalanced sample size is to assign a weight to the sample that is inversely proportionate to the class frequency. Since the weights are chosen with a fixed value to the number of samples of each class in the total sample, it does not work well for deep learning when using the batch gradient descent optimization method SGD. This is due to the overlap of features between different samples, as shown in Figure 1. As the number of samples increases, the features carried by new samples already exist in the original samples, and the model does not learn new features from the new samples, so this increase of sample size is ineffective for model training.

To address the problem of sample size imbalance, this paper rebalances the loss by effective samples size [18]. First, the effective sample size of each category is calculated using the following equation.

(1) $$\begin{array}{c} E_{n_{i}}=\frac{\;1-\beta^{n_{i}}}{1-\beta }, \end{array}$$

where *n*_*i*_ denotes the true number of samples in each category, *β* is the hyperparameter that controls the growth rate of *E*_*n*_*i*__ with *n*_*i*_, *β* ∈ (0, 1), and here, it is set at [0.9, 1). It can be seen from the above that a larger *E*_*n*_*i*__ indicates a larger effective sample size of category *i* in the training sample, and its loss proportion should be as small as possible. Therefore, the loss value is inversely related to the effective sample size as follows.

(2) $$\begin{array}{c} e_{i}=\frac{1}{E_{n_{i}}}=\frac{1-\beta }{1-\beta^{n_{i}}}. \end{array}$$

Secondly, considering the large difference in the number of each category, the effective sample size is normalized to get the sample size balance factor *α*_*i*_ for each category:

(3) $$\begin{array}{c} \alpha_{i}=\frac{e_{i}}{\sum_{j=1}^{k}e_{j}}=\frac{\left(1-\beta \right)/\left(1-\beta^{n_{i}}\right)}{\sum_{j=1}^{k}\left(\left(1-\beta \right)/\left(1-\beta^{n_{j}}\right)\right)}. \end{array}$$

where *k* denotes the number of categories. The weight *α*_*i*_ based on the effective sample size of each category is obtained from (3), and in turn, this weight is added to the loss calculation.

(4) $$\begin{array}{c} \text{Loss}=L\left(p\right)+\alpha_{i}L\left(p\right)=\left(1+\alpha_{i}\right)L\left(p\right), \end{array}$$

where *L*(*p*) denotes the original loss and *p* denotes the predicted probability. Here, *α*_*i*_*L*(*p*) is called the loss based on the effective sample size, and the total loss is the original loss plus the loss based on the effective sample size.

#### 3.1.2. Imbalance of Sample Difficulty

The difficult samples refer to less clearly classified borders on the transition region between the foreground and background, while the easy samples refer to background samples that do not overlap with the real target or positive samples that have a high degree of overlap with the real target. We proposed a method to determine and calculate the difficulty of samples. The basic idea is to calculate the distance between the prior probability distribution and the predicted probability distribution of a category and then measure the difficulty of the sample based on the magnitude of the distance.

First, the empirical class frequencies of each category [17] were calculated as their prior probabilities:

(5) $$\begin{array}{c} p_{p}\left(c_{i}\right)=\frac{{\left(1/n_{i}\right)}^{\rho }}{\sum_{j=1}^{k}{\left(1/n_{j}\right)}^{\rho }}, \end{array}$$

where *n*_*i*_ denotes the number of categories *c*_*i*_ and *ρ*, as a hyperparameter, denotes the degree of flexibility. After calculating the prior probability of each category, the prior distribution of the training samples is obtained. The cross-entropy function is then used to calculate the distance between the two distributions.

(6) $$\begin{array}{c} H\left(p_{p},p_{s}\right)=\overset{k}{\underset{i=1}{\sum }}-p_{p}\left(c_{i}\right)\log p_{s}\left(c_{i}\right), \end{array}$$

where *p*_*p*_ denotes the prior given matrix of the prior distribution and *p*_*s*_ denotes the matrix of each category of distribution obtained by the softmax function.

Considering the mutual exclusivity between categories in the classification problem, we only calculate the prior probabilities and predicted probabilities corresponding to the true categories in the two probability distribution matrices, where the true vector corresponding to a single category *c*_*i*_ is

(7) $$\begin{array}{c} {\text{true}}_{c_{i}}={\left[0,0,\cdots 1,\cdots 0\right]}^{T}. \end{array}$$

true_*c*_*i*__ is a *k*∗1 matrix. In this matrix, the value of the category *c*_*i*_ is 1 at the corresponding position, and the rest are 0. Next, we do the following calculation.

(8) $$\begin{array}{c} p_{p}^{T}*{\text{true}}_{c_{i}}=\left[p_{p}\left(c_{1}\right),p_{p}\left(c_{2}\right),\cdots ,p_{p}\left(c_{k}\right)\right]*\left[\begin{array}{c} \begin{array}{c} 0\\ 0 \end{array}\\ \cdots \\ \begin{array}{c} 1\\ \cdots \\ 0 \end{array} \end{array}\right]=p_{p}\left(c_{i}\right),\\ p_{s}^{T}*{\text{true}}_{c_{i}}=\left[p_{s}\left(c_{1}\right),p_{s}\left(c_{2}\right),\cdots ,p_{s}\left(c_{k}\right)\right]*\left[\begin{array}{c} \begin{array}{c} 0\\ 0 \end{array}\\ \cdots \\ \begin{array}{c} 1\\ \cdots \\ 0 \end{array} \end{array}\right]=p_{s}\left(c_{i}\right). \end{array}$$

In this way, we extract the individual category prior probability and the predicted probability, and this category must correspond to the true category, suppressing the interference of misinformation. In the following, a purer difficulty weight is obtained by calculating the distance between these two following the method in (6).

(9) $$\begin{array}{c} H\left(p_{p}^{T}*{\text{true}}_{c_{i}},p_{s}^{T}*{\text{true}}_{c_{i}}\right)=-p_{p}\left(c_{i}\right)\log p_{s}\left(c_{i}\right), \end{array}$$

where *p*_*p*_ denotes the prior probability for the category *c*_*i*_ and *p*_*s*_ denotes the predicted probability of the softmax output for the category *c*_*i*_.

#### 3.1.3. Double-Balanced Loss Function

The working principle of the double-balanced loss function is shown in Figure 2. In the classifier, the model obtains the prediction vector *Output* through the full connection layer, with the size of [3∗1], representing three kinds of lesions. Then, the model uses the softmax function to normalize this group of values, so that the probability vector *Prediction* of each model can be obtained. Before calculating the loss, the model calculates the quantity weight and the difficulty weight according to equations (4) and (9), respectively. Based on these two weights, the double-balanced loss calculates the distance between the predicted value (Prediction[3∗1]) and the true value as the final loss value, and this loss value is used as a feedback signal passed to the optimizer, and then, the optimizer implements the neural network weight update through the back propagation algorithm.

In this paper, we use cross-entropy as the original loss, which is responsible for calculating the difference between the true value and the predicted value, and use the one-hot coding in the calculation to obtain a concise expression:

(10) $$\begin{array}{c} {\text{CE}}_{\text{loss}}=-\log p_{s}. \end{array}$$

Bringing (10) into (4) yields the loss based on the effective sample.

(11) $$\begin{array}{c} \text{los}{\text{s}}^{\prime }=-\left(1+\alpha_{i}\right)\log p_{s}. \end{array}$$

Then, the formula for calculating the difficulty weights in (9) is added to (11), and the double-balanced loss function can be obtained as follows.

(12) $$\begin{array}{c} {\text{DB}}_{\text{loss}}=\left(1+\frac{\left(1-\beta \right)/\left(1-\beta^{n_{i}}\right)}{\sum_{j=1}^{k}\left(\left(1-\beta \right)/\left(1-\beta^{n_{j}}\right)\right)}\right)\left(\frac{{\left(1/n_{i}\right)}^{\rho }}{\sum_{j=1}^{k}{\left(1/n_{j}\right)}^{\rho }}\right){\left(\log p_{s}\right)}^{2}, \end{array}$$

where *β* and *ρ* are hyperparameters, *k* is the number of categories, and *n*_*i*_ is the number of training samples corresponding to category *i*.

### 3.2. Materials

The dataset used in this paper was obtained from white-light endoscopy images of patients' colonoscopy, provided by the Gastrointestinal Endoscopy Center of the East Hospital of Shanghai Sixth People's Hospital. We named this dataset SSPH_WL. The SSPH_WL was collected by doctors under ethical approval. The colorectal lesions were classified into three categories (polyp, adenoma, and cancer) in combination with clinical diagnosis. Sample images of the three categories are shown in Figure 3.

The dataset was collected from June 2015 to September 2019, and a total of 1709 white-light endoscopic images containing lesions were collected and labeled by physicians with more than 5 years' clinical diagnostic experience in gastroenterology endoscopy. Among them, there were 1048 adenomatous cases, 381 polypoid cases, and 280 cancerous cases. The SSPH_WL was divided into the training set (SSPH_WL-I) and test set (SSPH_WL-II) according to 8 : 2.

We also use colorectal white-light endoscopic images from the public datasets CVC_ClinicDB [23], CVC_ColonDB [24], and Kvasir [25] as the test sets to further evaluate the generalization ability of the classification model. 428 colonoscopic images are selected from the Kvasir data, including 180 images of adenoma, 73 images of cancer, and 175 images of polyp. 95 images are selected from CVC_ClinicDB, CVC_ColonDB and our collection of videos, including 36 images of polyp and 40 images of adenoma, and 19 images of cancer from colorectal cancer videos, named CVC. All of the above datasets were annotated by experienced gastroenterology endoscopy clinicians. The detailed descriptions of these three datasets are shown in Table 2.

## 4. Experimental Results and Discussion

### 4.1. Training Strategy and Evaluation Metrics

Deep learning-based object detection models can be divided into two categories: two stage and one stage. Due to the complex background of the gut, the two-stage algorithm performs background filtering first to overcome this problem, so we choose the two-stage object detection model Faster R-CNN [8] as the representative and focus on the classification effect of the double-balanced loss in this model. The momentum is set to 0.9; the initial learning rate (lr) is 0.005 and automatically decreases by two-thirds every three epochs. For other parameters, we use the default values in the model. For the backbone feature extraction network, we choose ResNet50 based on natural image pretraining, which can make the initial performance of the model higher and converge faster by assisting us to train the model through transfer learning. As shown in Figure 4, Since the loss value no longer decreases, the model reaches the optimum at this time and stops training.

This study is a multilabel classification, and the accuracy is not suitable for evaluating the performance of a model for a single category due to the data imbalance. This paper uses AP and AR as model evaluation indicators. AP (Average Precision) is the area under the P-R curve and can be used to measure the performance of the model for a single category, and AR represents the average recall rate of the classification. These two indicators can be expanded as follows.

AP : AP at IoU = 0.50 : 0.05 : 0.95.

AP_50_ : AP at IoU = 0.50.

AP_75_ : AP at IoU = 0.75.

AR : AR given 1 detection per image.

AR_10_ : AR given 10 detections per image.

AR_100_ : AR given 100 detections per image.

IoU (Intersection-over-Union) represents the ratio of the intersection and the union of the predicted border and the ground truth bound. In addition, we add the missed detection rate (False Negative Rate, FNR) and the wrong detection rate (False Positive Rate, FPR), which are common evaluation indicators for computer-aided diagnosis. These two indicators are calculated as follows.

(13) $$\begin{array}{c} \text{FNR}=\frac{\text{FN}}{\text{TP}+\text{FN}}, \end{array}$$

(14) $$\begin{array}{c} \text{FPR}=\frac{\text{FP}}{\text{FP}+\text{TN}}. \end{array}$$

In equations (13) and (14), TP is true positive, TN is true negative, FP is false positive, and FN is false negative.

### 4.2. Experiment on Hyperparameter

The double-balanced loss function has two parameters, where *β* is responsible for regulating the effective sample size and *ρ* is responsible for regulating the prior probability of the category. Usually, *β* ∈ [0, 1); in this paper, the number of training samples of each category is {adenoma = 838, cancer = 224, polyp = 305}, and when *β* ∈ [0, 0.9), the three effective sample sizes calculated from the training samples are almost equal, and the difference of sample sizes cannot be reflected at this time, so *β* ∈ [0.9, 1) is set. As shown in Figure 5, starting from *β* = 0.99, the difference of the effective sample size corresponding to the three categories starts to appear, and as *β* increases, the effective sample size is closer to the true number. For the parameter *ρ*, since the number of each category in the training data is fixed, when *ρ* = 0, it means that each category has the same prior distribution, and when *ρ* = 1, it is equivalent to each category having a prior distribution based on the inverse class frequency.

As shown in Figures 6(a)–6(c), the change curve of the weighted value of the loss function with the prediction probability, looking at each line alone, there is a trend: the higher the predicted probability, the smaller the weighted value, which means that the loss of simple samples is suppressed; looking at the three category curves, the weighted value of adenoma with the largest number of samples is always the smallest, which means that the loss of the multisample category is suppressed. In Figures 6(a) and 6(b), when *β* is constant, the larger *ρ* is and the larger the weighted gap between the three categories. In Figures 6(a) and 6(c), when *ρ* is constant, the larger *β* is, the larger the weighted gap between the three categories will also be. By adjusting hyperparameter *β* and *ρ*, the model forms a dynamic weighting mechanism of loss function during training, which can make the model update parameters in a more reasonable way.

In this paper, the comprehensive experiments are conducted for the parameter values, and the corresponding results of different parameter values are shown in Table 3. From the overall performance, the average precision and average recall of detection are almost optimal for *β* = 0.99 and *ρ* = 0.25, so we mainly conduct experiments under this parameter value.

### 4.3. Improved Results on Faster R-CNN

The original loss function used for classification in Faster R-CNN is cross-entropy (CE) loss. Thus, comparing the CE loss, it is clear to see the improvement brought by the DB loss. The training set SSPH_WL-I and test set SSPH_WL-II are from the dataset SSPH_WL, so their data distribution are the same.  Figure 7 shows the AP_50_ (IoU = 0.5) changes with epoch on SSPH_WL-II; DB loss can help the model steadily improve the AP_50_ value, where the AP_50_ using the DB loss in Faster R-CNN is stable at around 0.850 and up to 0.858, and the AP_50_ using the CE loss is stable at around 0.820 and up to 0.824.  Table 4 compares the detection results of the one-stage model SSD [26]; for the colorectal polyp lesion detection, Faster R-CNN performs better than SSD, and the use of double-balanced loss function can significantly improve the detection performance of Faster R-CNN and SSD.

Table 5 shows a comparison of the results on SSPH_WL-II, Kvasir, and CVC. In these three test sets, DB loss achieves a great lead in all metrics. Kvasir and CVC are used as additional test sets to verify the generalization of DB loss, and the results show that Faster R-CNN trained based on DB loss has a good generalization ability.

In our study, we focus not only on the overall classification level of the model but also on the model's ability to distinguish the three categories.  Figure 8 shows the comparison of the classification effect (AP_50_) of the model on the three test sets. On SSPH_WL-II, the model has the worst classification effect on polyp, and after improvement, the classification precision of polyp is improved the most. On Kvasir and CVC, the model has the worst classification effect on cancer, and after improvement, the classification precision of cancer is improved the most. This indicates that the model can focus on the samples that are not good at classification after improvement, and the classification precision of the three categories is balanced in this way.

We use three test sets to further evaluate the classification ability of the model in terms of the wrong detection rate (FPR) and the missed detection rate (FNR). The wrong detection refers to the model that can locate the lesions but cannot classify them correctly. This is caused by the insufficient classification ability of the model. The missed detection refers to lesions that are not detected by the model, which are filtered out mainly because the model does not locate the lesion or the classification confidence is lower than the set threshold. As shown in Table 6, the FPR and FNR have decreased by using DB loss, indicating that the classification ability of the model has been improved.

The confusion matrices are shown in Figure 9. For the wrong detection, in the original model, 18 adenomas are wrongly classified as cancer, 7 cancers are wrongly classified as adenoma, 11 adenomas are wrongly classified as polyp, and 7 polyps are wrongly classified as adenoma; after using the double-balanced loss, 10 adenomas are wrongly classified as cancer, 6 cancers are wrongly classified as adenoma, 6 adenomas are wrongly classified as polyp, and 6 polyps are wrongly classified as adenoma. It is not difficult to find that the wrong detection never occurs between cancer and polyp; this is due to the huge difference in characteristics between polyp and cancer.

In addition, some disturbances in the intestine may also lead to wrong detection of the model, as shown in Figure 10 There are three main categories of these disturbances: the first is the identification of the reflected light spots in the intestine as lesions, the second is the identification of foreign matter in the intestine as lesions, and the third is the identification of air bubbles in the intestine as lesions.

As for missed images, DB loss reduces the occurrence of missed detection, but there are still missed detections, as shown in Figure 11. Most of these images are characterized by small target areas, dim light, and occlusion, which may be the main reason for missing model detection.

### 4.4. Comparison Experiments of Different Loss Functions

We compare the classification effects of weight cross-entropy loss (WCE), multiclassification focal loss (FL), and class-balanced cross-entropy (CB) loss in Faster R-CNN, all of which can be used to solve the imbalance problem.

As shown in Table 7, the classification effects of different loss functions on different test sets are compared. On SSPH_WL-II, the double-balanced loss achieves the advantage in all metrics, and on Kvasir, the double-balanced loss and the class-balanced cross-entropy loss perform the best. On CVC, these four loss functions achieve better results, and the double-balanced loss function comes out ahead in all metrics. Experiments show that the double-balanced loss has good generalization ability on different test sets and is able to solve the data imbalance problem better than other loss functions.

Comparing the classification effects of weight cross-entropy (WCE), multiclassification focal loss (FL), and class-balanced cross-entropy (CB) loss functions in Faster R-CNN, as shown in Figure 12, we can see that the double-balanced loss function proposed in this paper has the following advantages: in example (a), the classification is more accurate; in example (b), the classification confidence is higher; and in example (c), the classification performance is better for small targets.

## 5. Conclusions

To address the imbalance problem in medical image classification, this paper proposes a new loss function, namely, the double-balanced loss. This loss function improves the classification ability of the model for this part of samples by increasing the focus on fewer sample categories and difficult samples during model training. In this paper, we mainly achieve the double-balanced loss function in Faster R-CNN, and after three test set validations, the model achieves the best detection effect at IoU = 0.5, when the AP values are improved by 3.4%, 8.3%, and 2.9%, indicating that the double-balanced loss function achieves the expected effect on the classification of colorectal white-light endoscopic images. However, there are various types of medical images, and we will verify the effectiveness of the double-balanced loss function on other imbalanced datasets and further promote the double-balanced loss function in the next work.

## Figures and Tables

**Figure 1:** The features contained in the new samples may already be partially or fully contained in the original samples.

**Figure 2:** Double-balanced loss working principle, balancing loss in terms of both sample size and sample difficulty.

**Figure 3:** White-light endoscopy images of patients' colonoscopy: (a) adenoma, (b) polyp, and (c) cancer.

**Figure 4:** Loss variation curves for training: yellow curve represents RPN loss and blue curve represents classifier loss.

**Figure 5:** The effective sample size changes with the hyperparameter *β*.

**Figure 6:** Analysis of *β* and *ρ*. Variation curve of weight.

**Figure 7:** The AP50 (IoU = 0.5) changes with epoch on SSPH_WL-II by using CE and DB.

**Figure 8:** Comparison of classification effect by using CE and DB: (a) cross-entropy loss; (b) double-balanced loss.

**Figure 9:** Confusion matrix: (a) cross-entropy loss function; (b)double-balanced loss function.

**Figure 10:** Three main categories of disturbances: (a) light spot, (b) foreign matter, and (c) bubble.

**Figure 11:** Missed detection images of three test datasets.

**Figure 12:** Comparison of different loss function detection results. True category is (a) adenoma, (b) cancer, and (c) polyp.

**Table 1:** Deep learning in the diagnosis of colorectal white-light endoscopy.

Study	Date	Model	Classes
Komeda et al. [3]	2016	CNNs	Neoplastic, nonneoplastic
Eduardo et al. [4]	2017	CNNs	Adenoma, nonadenoma
Gao et al. [5]	2020	Mask R-CNN	Cancer, adenoma, polyp
Taş and Yilmaz [7]	2021	Faster R-CNN	Polyp, nonpolyp
Shin et al. [9]	2018	Faster R-CNN	Polyp, nonpolyp
Shin et al. [10]	2019	Faster R-CNN	Polyp, nonpolyp
Nogueira-Rodríguez et al. [11]	2020	YOLO	Polyp, nonpolyp

**Table 2:** The datasets used in this experiment: SSPH_WL-I is used for training, SSPH_WL-II, Kvasir, and CVC is used for test.

Dataset	Used for	Description	Resolution (*w* × *h*)	Public
SSPH_WL-I	Train	1367 images	375 × 347	No
SSPH_WL-II	Test	342 images	375 × 347	No
Kvasir	Test	428 images	Various resolutions	Yes
CVC	Test	95 images	388 × 284 574 × 500	Yes

**Table 3:** AP and AR of Faster R-CNN with different parameter values.

*β*	*ρ*	AP	AP_50_	AP_75_	AR	AR_10_	AR_100_
0.9	0.25	0.578	0.854	0.678	0.669	0.718	0.718
0.99	0.25	0.598	0.858	0.712	0.675	0.731	0.733
0.999	0.25	0.585	0.858	0.696	0.672	0.710	0.711
0.9999	0.25	0.57	0.833	0.694	0.656	0.707	0.707
0.9	0.5	0.587	0.853	0.695	0.662	0.717	0.717
0.99	0.5	0.582	0.838	0.7	0.671	0.726	0.726
0.999	0.5	0.582	0.843	0.675	0.653	0.715	0.716
0.9999	0.5	0.571	0.826	0.679	0.661	0.709	0.709
0.9	0.75	0.579	0.852	0.663	0.669	0.718	0.718
0.99	0.75	0.562	0.836	0.627	0.654	0.704	0.704
0.999	0.75	0.584	0.85	0.667	0.675	0.713	0.714
0.9999	0.75	0.597	0.848	0.717	0.674	0.719	0.719

**Table 4:** Comparison of the improvement effects of Faster R-CNN and SSD on SSPH_WL-II.

Model	Loss	AP_50_	AR_100_
Faster R-CNN	DB	0.858	0.733
Faster R-CNN	CE	0.824	0.711
SSD	DB	0.835	0.701
SSD	CE	0.821	0.689

**Table 5:** Comparison of the improvement effects of Faster R-CNN on three test sets.

Dataset	Loss	AP	AP_50_	AP_75_	AR	AR_10_	AR_100_
SSPH_WL-II	DB	0.598	0.858	0.712	0.675	0.731	0.733
	CE	0.564	0.824	0.638	0.660	0.711	0.711

Kvasir	DB	0.528	0.833	0.552	0.601	0.661	0.661
	CE	0.475	0.750	0.505	0.594	0.652	0.652

CVC	DB	0.639	0.948	0.745	0.677	0.770	0.770
	CE	0.583	0.874	0.649	0.656	0.698	0.698

**Table 6:** Wrong detection rates and missed detection rates.

Loss	FPR	FNR
DB	3.24	3.01
CE	4.97	3.47

**Table 7:** Performance of different loss functions on the three test sets.

Dataset	Loss	AP	AP_50_	AP_75_	AR	AR_10_	AR_100_
SSPH_WL-II	DB	0.598	0.858	0.712	0.675	0.731	0.733
	WCE	0.577	0.842	0.669	0.658	0.724	0.724
	FL	0.571	0.813	0.662	0.667	0.719	0.719
	CB	0.574	0.834	0.681	0.661	0.728	0.726

Kvasir	DB	0.528	0.833	0.552	0.601	0.661	0.661
	WCE	0.458	0.764	0.459	0.581	0.637	0.637
	FL	0.453	0.739	0.459	0.581	0.639	0.639
	CB	0.500	0.788	0.570	0.605	0.661	0.661

CVC	DB	0.639	0.948	0.745	0.677	0.770	0.770
	WCE	0.593	0.885	0.668	0.662	0.705	0.705
	FL	0.597	0.864	0.668	0.663	0.711	0.712
	CB	0.619	0.905	0.676	0.672	0.735	0.735

## Data Availability

The data used to support the findings of this study are available from the corresponding author upon request.
